The article "Radiographic Diagnosis of Fibrous Dysplasia in Maxilla" was published in 2018. Journal: Cureus.

# Radiographic Diagnosis of Fibrous Dysplasia in Maxilla

**DOI:** 10.7759/cureus.3127

**Published:** 2018-08-10

**Authors:** Natalie E Kochanowski, Mahmoud S Badry, Ahmed Z Abdelkarim, Scott Lozanoff, Ali Z Syed

**Affiliations:** 1 Pre-Medical School, University of Hawaii at Manoa, Honolulu, USA; 2 Oral and Maxillofacial Radiology, British University, Cairo, EGY; 3 Anatomy, Biochemistry & Physiology, University of Hawaii School of Medicine, Honolulu, USA; 4 Oral Medicine and Diagnostic Sciences, CWRU School of Dental Medicine, Cleveland, USA

**Keywords:** fibrous dysplasia, ground glass, mixed radiopacity, cbct

## Abstract

Fibrous dysplasia is a rare bone disorder characterized by the replacement of normal bone by abnormal fibrous tissue. Here we present a 16-year-old female with a fibrous dysplasia in the maxilla and obliteration of the sinus in the same side. Cone beam computed tomography scan revealed a mixed radiopacity that extended from the alveolar crest of the right posterior teeth to the right orbital floor in the superior-inferior direction. The radiopaque areas had homogenous ground glass appearance. There is a loss of bone trabeculation, thinning of the cortical boundaries but still intact, and a loss of the lamina dura around the right posterior permanent teeth. The radiographical features of the lesion were indicative of fibrous dysplasia in the maxilla.

## Introduction

Fibrous dysplasia is a rare bone disorder characterized by the replacement of normal osseous tissue by abnormal fibrous tissue. This disorder was first discovered by Lichtenstein in 1938, who later collaborated with Jaffe in 1942 to first describe the condition in the medical literature [1]. The replaced bone showed the trabeculae as shorter, thinner, irregularly shaped, and more numerous [2]. It was determined that the abnormal appearance of the bone corresponds to increased weakness and expansion that may further lead to bone deformation and possible fractures. This abnormal bone disorder may occur alongside a condition known as McCune-Albright syndrome. This disorder is caused by a GNAS1 point mutation on chromosome 20 [3]. These changes inhibit GTPase activity that is normally required to deactivate the G protein, thereby altering signal transduction pathways. The increased amount of cAMP in bone stromal cells leads to unregulated proliferation and differentiation [4].

Fibrous dysplasia may be sub-categorized as either monostotic, in which case only one bone is affected, or polyostotic, in which two or more bones are affected [5]. These forms most commonly affect regions of the ribs, femur, and the craniofacial region. The extent of this case report will focus on the bones found in the craniofacial zone, i.e., mandible, maxilla, zygoma, and temporal bones that can be affected in either monostotic or polyostotic forms [6]. Monostotic bone replacement is more common in the posterior portion of the maxilla, occurring almost twice as often compared to the mandible [7].

The article "Radiographic Diagnosis of Fibrous Dysplasia in Maxilla" was published in 2018. Journal: Cureus.

The monostotic form of fibrous dysplasia is usually found in older age groups while the polyostotic form is associated with children under the age of 10 years [2]. Moderate symptoms of the disease include swelling and enlargement of craniofacial regions. However, when the disease progresses without diagnosis and treatment, it can lead to loss of vision, hearing, airway obstruction, anosmia, and numbness [8]. Fibrous dysplasia of the maxilla or mandible may cause the displacement of permanent teeth, interfere with the eruption of new teeth, and contribute to malocclusion [9]. In most cases, bone dysplasia is diagnosed incidentally as a result of facial asymmetry, facial distortion/deformity, and radiological images [7]. Confirmation of craniofacial fibrous dysplasia is achieved through image analysis of plain radiographs, magnetic resonance images, or computed tomographic images as well as biopsy. There is no cure for fibrous dysplasia currently, but treatment is capable of diminishing the effects of symptoms. Various bisphosphonates are administered in an attempt to prevent further bone loss [5]. If bone fractures occur from fibrous dysplasia, then surgical intervention is frequently required. Surgery focuses on removing connective tissue to restore normal facial aesthetics but is often unable to reverse complications in the orbital, nasal, and temporal regions.

A computed tomography (CT) scan and magnetic resonance imaging (MRI) may be able to further confirm the presence and severity of the disease following initial observations derived from a standard X-ray. Among these imaging techniques, there are key features that are examined in order to more easily identify the presence of fibrous dysplasia. The abnormal growth of lesions can often be identified as either radiolucent or radiopaque or a mixture of both [2]. The innermost border of the maxilla and skull usually contain radiopaque features without distinct borders. These characteristics may be further divided into various categories of internal bone patterns. Four distinct bone patterns are as follows: 1) fingerprint-like pattern, 2) granular pattern, 3) cotton-wool pattern, and, 4) orange-peel pattern [2]. The identification of these patterns enable a better understanding of the extent and depth of the lesion, facilitating a more specific diagnosis.

## Case presentation

A 16-year-old female presented in a private dental clinic with a chief complaint of pain and swelling on the right maxillary side. Upon intra-oral examination, a bony swelling was noticed in the right buccal vestibule. The patient was then referred to a private dental imaging center for imaging of the jaws to determine the presence and extent of the lesion. A cone beam computed tomography (CBCT) scan was taken for the area of interest.

The article "Radiographic Diagnosis of Fibrous Dysplasia in Maxilla" was published in 2018. Journal: Cureus.

A board-certified oral and maxillofacial radiologist performed the radiographic interpretation of the CBCT scan. The scan revealed a mixed radiopacity in the right side of the maxilla. Sagittal cuts show that the lesion extended from the alveolar crest of the right posterior teeth (from the first premolar to the third molar and pterygoid plates) to the right orbital floor in the superior-inferior direction (Figure 1).

**Figure 1:** Sagittal view showing the extension of the lesion anteroposteriorly and superior-inferiorly (yellow circle).

Axial cuts revealed that the lesion obliterated the right maxillary sinus completely and caused expansion of the anterior, posterior, and lateral walls of the right maxillary sinus while maintaining the maxillary sinus outline (Figure 2).

**Figure 2:** Axial view showing the extension of the lesion mediolaterally, obliteration of the right maxillary sinus with lateral and anterior walls expansion (yellow arrows).

Coronal cuts showed that the lesion extended from the lateral wall of the right nasal cavity to the lateral wall of the right maxillary sinus and zygomatic arch with expansion in both lateral and superior walls of the maxillary sinus (Figure 3).

**Figure 3:** Coronal view showing complete obliteration of the right maxillary sinus by the lesion with superior expansion of the lesion toward the orbit and in lateral direction towards the zygomatic arch, (yellow arrows).

The lesion blended with the surrounding normal bone, and the internal structure showed mixed radiopaque-radiolucent areas characterized by a homogenous “ground glass” appearance (Figure 4).

**Figure 4:** Axial view showing the nature of the lesion. The mixed radiolucent-radiopaque lesion blends with the surrounding structures (yellow circle).

Additional observations included a loss of bone trabeculation, thinning of the cortical boundaries, and a loss of the lamina dura around the right posterior permanent teeth (Figure 5). Differential diagnosis included ossifying fibroma, fibrous dysplasia, and osteomyelitis. Based on the radiographic features such as anatomical expansion, lack of root resorption, lack of onion skin appearance, an impression of fibrous dysplasia was made. In our case no aggressive surgical treatment was planned because of recurrence during the active growth phase.

The article "Radiographic Diagnosis of Fibrous Dysplasia in Maxilla" was published in 2018. Journal: Cureus.

**Figure 5:** A sagittal view showing the thinning in the cortical boundaries of the lesion without loss of integrity (yellow arrows). A loss of lamina dura of the right posterior permanent teeth is evident (red arrows).

## Discussion

The age of the patient indicates that younger individuals are more likely to present with fibrous dysplasia. In fact, polyostotic fibrous dysplasia most commonly occurs in children under 10 years of age. In most cases, the lesions proliferate in the craniofacial region of these young patients, in prepubescent patients, but slows and stabilizes during puberty [3]. Although the onset may begin at a young age, the disease is not diagnosed and treated until the teenage years.

The craniofacial region is involved in 90% of fibrous dysplasia cases and typically localizes to the zygomatic-maxillary complex rather than the mandible [8]. This pattern was present in the current case report with scans revealing the expansion of the maxillary sinus.

As observed in Figure 4, the radiolucent-radiopaque pattern is a result of the lesions transforming from a “ground glass” appearance to a mixed appearance as adulthood approaches [8]. The mixed appearance of the lesion results in ‘blending’ due to the absence of a distinct edge. The appearance of a homogenous pattern can be attributed to the loss of lamina dura. In a similar case study, a radiograph revealed loss of lamina dura surrounding premolar and molar teeth with granular radiopacities in the periapical areas [10]. The obliteration of the maxillary sinus is thereby due to the presence of the lesion, which blends with its boundaries.

Surgical treatment of fibrous dysplasia could be either a conservative approach by shaving or contouring the bone or radical excision followed by reconstruction [11]. The choice of the surgical option depends on several factors such as site of involvement, patient preference, and the availability of a multidisciplinary team. Medical treatment has a role in the management of craniofacial fibrous dysplasia. Some authors have reported their experience with the use of steroids, mainly in the treatment of visual symptoms from optic nerve compression [6].

## Conclusions

Fibrous dysplasia is a rare bone disorder characterized by the replacement of normal osseous tissue by abnormal fibrous tissue. CBCT is an informative modality to further confirm the presence and severity of the disease following initial observations derived from a standard X-ray.
